# Cultivation and interpretation of students' psychological quality: Vocal psychological model

**DOI:** 10.3389/fpubh.2022.966628

**Published:** 2022-07-29

**Authors:** Yali Zhang

**Affiliations:** Anyang Normal University, Anyang, China

**Keywords:** vocal music teaching, student expressiveness, mental health, simulation model, data mining

## Abstract

Reflecting students' mental health data through vocal music teaching expressive system is a research hotspot in vocal music teaching psychology. Based on the theory of students' expressiveness in vocal music teaching, this paper constructs a psychological model of vocal music teaching. The model uses psychological data mining technology to conduct a feasibility study and analysis on the mental health education of vocal music students, solves the quantitative problem of mental health, and analyzes the relationship between psychological problems and students. In the simulation process, the psychological data of the vocal music freshmen of a certain college was taken as the research object, and the association rule Apriori algorithm was used to analyze the relationship between the factors of the psychological dimension. Psychological data mining was carried out, and descriptive indicators and univariate analysis methods were used to analyze the current situation of students' mental health and personality characteristics, and Pearson correlation analysis and structural equation model were used to explore the relationship between their mental health and personality characteristics. The amount of vocal music learning is the duration of the load and the total number of tasks completed within a single exercise or a series of exercises. ASP-NET and SQLServer2008 and other experimental results show that the chi-square test value of the overall fit of the model is 20.078, and the ratio of the chi-square value to the degree of freedom is 4.016, which has a relatively high accuracy and effectively enhances the psychological data mining technology in vocal music students for operation and practicality of applications in health data analysis.

## Introduction

With the deepening of vocal music theory research, interdisciplinary knowledge is further infiltrating into the practice of vocal music teaching (1). Due to the particularity of vocal music teaching, the bridge between vocal music teaching and vocal music knowledge is getting closer and closer (2), we continue to develop and attach importance to vocal music knowledge in the process of learning and vocal music teaching, and gradually become a benchmark in the field of vocal music and even art (3), so the development and utilization of vocal music knowledge is the pace of the times, it can improve students' second-degree creation ability and understanding and expression ability of works, and it is also conducive to cultivating students' emotions, attitudes and values (4–6). In vocal music teaching, the smooth communication between teachers and students and students' learning attitude directly affects their singing performance, so the research on vocal music knowledge is an important way to improve the efficiency of vocal music teaching (7).

Personality characteristics refer to the stable psychological characteristics gradually formed by individuals in the process of psychological development. The formation of personality traits is closely related to environmental, educational, social and genetic factors (8). A person's personality traits have a great impact on their psychological characteristics and behavior. Mental health refers to an individual's ability to adapt to the current and developing environment, to have complete personality characteristics, to be in a positive state of cognition, emotional response, and volitional action (9–11), and to maintain a normal ability to regulate. Personality characteristics refer to the stable psychological characteristics gradually formed by individuals in the process of psychological development. A person's personality characteristics have a great influence on their psychological characteristics and behavior (12). Vocal music students work in a special natural and social environment, and it is of great significance to study their mental health status and personality characteristics, as well as the relationship between the two, to implement mental health education and improve the mental health level of vocal music students (13).

This paper uses the literature of vocal music psychology, pedagogy and other fields as theoretical basis, combined with years of vocal music singing and vocal music teaching practice, to make a preliminary research on a large amount of vocal music knowledge in vocal music learning. In the initial stage of designing the mental health assessment system for vocal music students, the first task is to organize the design of the system architecture. In order to stabilize the use of psychological assessment and avoid network congestion when students visit at the same time, the method of participating in different majors and batches is adopted. The system and psychological data are separated and deployed on different servers. The two servers assume different functional roles. The concurrent processing capability of the system and the storage space of psychological data are well guaranteed. The 90-scale questionnaire and the 16PF personality factor questionnaire were provided by the college; descriptive indicators and univariate analysis methods were used to analyze the current situation of occupational divers' mental health and personality characteristics, and Pearson correlation analysis and structural equation model were used to explore their psychological status. After calculating the results of these two indicators that affect the psychological load of students in vocal music class, they are weighted according to their respective weights to obtain the final psychological load value of students in vocal music class. The scale can comprehensively reflect all aspects of mental health, and is recognized as the first scale for evaluating mental health. It has good validity and reliability. In the classification and diagnosis of mental health symptoms, it can reflect the physical and mental stress of vocal music students. The status and existing psychological problems can be used as an assessment tool to detect various types of neuroses, and can be used in psychological counseling and mental health evaluation.

## Related work

The study found that the layered vocal music teaching had a positive impact on the students' previous habitual learning process and methods, making students' learning more confident and goal-oriented, enabling students at different levels to improve on the original basis, and making them more confident. The gap between students at different levels has been reduced (14). After researching the current specific vocal music teaching links, it was found that self-efficacy is the most important factor affecting academic performance, and students' listening time in class is the core factor (15).

First of all, in terms of congenital factors, Clifford (16) found through investigation that gender difference is not an influencing factor of academic achievement in vocal music. In different grades, gender difference does have an impact on the academic achievement of eighth-grade students, but it is not significant. After adding geographical factors, gender differences in vocal music academic achievement are greater in suburbs than in urban areas. In the research on visual perception ability, Heyman's (17) research shows that this is one of the influencing factors of academic achievement in vocal music. Training visual perception ability can effectively improve vocal performance, and it is more effective for students with poor visual perception ability. Knapp (18) found that the spatial ability of visual perception can affect the development of vocal symbolic awareness, and through the neural level symbolic awareness as a medium to affect the visual level symbolic awareness, thereby affecting the academic achievement of vocal music.

Zhou (19) conducted a study on students' learning styles and found that factors such as learning confidence and learning expectations have an impact on their academic achievement, and found that cognitive strategies and metacognitive strategies can have a significant impact on vocal academic achievement, students' learning styles are divided into divergent thinking type, convergent thinking type, adaptive type and absorption type, and then study the influence of cognitive strategy, resource management strategy and metacognitive strategy. Obviously, it has little effect on resource management strategies of convergent thinking and adaptive students, and has little effect on cognitive strategies of absorbing students (20). Similarly, there are some influencing factors that change with academic performance or age, such as the self-concept mentioned above, as well as other such as non-symbolic quantitative representation ability and symbolic awareness (21). The researchers found that the approximate number system, as one of the innate number systems of human beings, is not significantly related to the academic performance of vocal music at the beginning of children's formal vocal music education (22). More complex, the relationship between approximate number systems and vocal performance has gradually become significantly correlated (23, 24).

## Construction of vocal music teaching psychological model based on cultivation and interpretation of students' expressiveness

### Hierarchical equation of vocal expressiveness

Vocal expressiveness hierarchical classification rules use the training set to establish a classifier or model to classify psychological data; association rules need to find frequent itemsets from each psychological database transaction, that is, all itemsets whose support degree g(x) is greater than the minimum support degree, and then filter out association rules are rules that satisfy both minimum support and minimum confidence. Although the error of parameter estimation is often large in the initial stage of iteration, the fitting function is also very large; but as the number of iterations increases, the parameter estimation value becomes more and more accurate, and the fitting function gradually converges to the minimum value x. If the iteration does not converge, the model u has no solution; there are many missing values or outliers in the psychological data y-x and improper model selection can lead to the non-convergence of the iteration xr(x,y).


(1) $$G_{i}(x)=\langle \begin{array}{c} 20+70(1-2x-t),x>t\\ 10-50(1.2+3x+4t),x<t \end{array}$$

(2) $$\begin{array}{c} xr(up,x,y)=\left[\begin{array}{c} F_{i}(x-u,x+u)\\ F_{i}(y-x,y+x) \end{array}\right] \end{array}$$

After the psychological data is uniformly coded, it is entered into the EXCEL psychological database. First, apply SPSS10.0 statistical software package to SCL 90 and 16PF scores were used for basic statistical analysis; on this basis, LISREL8.53 was used to further analyze the relationship between the two. Among them, cs(i,j) is the endogenous latent variable; fix(i) is the exogenous latent variable; r is the coefficient matrix of the palm in the mxn order structural relationship, reflecting the influence of the exogenous latent variables on the endogenous latent variables; cos(i) is the residual term of the structural equation, that is, the vector formed by the error of the structural equation between the order and fix(i), reflects the unexplained part of f(x) in the equation.


(3) $$\begin{array}{c} F_{i}(x,cs(i,j))=\left[\begin{array}{c} fix(i-j)-i\\ fix(i-1)-i-1\\ fix(i-cs)-x \end{array}\right] \end{array}$$

(4) $$\begin{array}{r} \underset{i,j=1}{\sum }x^{t-i}\left(i\right)/\cos{\left(x\right)}^{t-j}\left(j\right)=\underset{i,j=1}{\sum }\cos^{t-i}\left(i\right)/x^{t-j}\left(j\right)-\cos\left(i,j\right) \end{array}$$

Among them, sign(x) is the endogenous index, that is, the vector composed of the pxl-order endogenous observation variables; x is the exogenous index, that is, the vector composed of the q × pi-order exogenous observation variables; pin is the exogenous index x, that is, the vector formed by the measurement error of q × 1 order x.


(5) $$\begin{array}{r} g\left(x,sign\left(x\right)\right)=\left(sign\left(is\right)-sign\left(j\right)\right)-gx\left(i\left(s\right)/i\left(t\right)-1\right) \end{array}$$

(6) $$\cos(\frac{x}{2pin},sign(x))=\{\begin{array}{c} \cos(2i-pin)\\ \left(sign(is)-\frac{x}{2pin})(2pi-1\right) \end{array}$$

The ratio of the chi-square value to the degrees of freedom is 0.615, the psychological data is low, and the significant probability value *p* = 0.541 > 0.05, so the null hypothesis is accepted, so it is assumed that the model can fit the observed psychological data. The GFI value, AGFI value and CFI value are all high, the CFI value is even 1, and the RMSEA value is 0, so the model observation psychological data is completely fit. Therefore, the reliability of the above model is good, which means that the above-mentioned observation variables affect the academic mood of high school students, which in turn affects their academic achievement in vocal music. The mean and standard deviation or the median and quartile are used to describe the mean level and discrete trend of the scores: due to the large sample size of this data (*m* = 70), when the vocal students are compared with the norm, the single-sample numerical variables are used, comparisons of constituent ratios use row × column z2 test and multiple comparisons between multiple sample rates in Table 1, to apply linear correlation to analyze the relationship between SCL-90 and 16PF scores.

**Table 1:** Vocal expressiveness hierarchy.

**Vocal case**	**Questionnaire value**	**Content validity**	**Construct validity**	**Chi-square value**
10	42	0.87	0.35	0.79
20	83	0.40	0.72	0.65
30	57	0.45	0.43	0.01
40	56	0.77	0.76	0.12
50	99	0.43	0.43	0.98
60	66	0.11	0.88	0.28
70	63	0.12	0.99	0.36

The validity of the questionnaire was tested by content validity and construct validity. For the content validity analysis, five experts were invited to evaluate the content validity of each item, and the scoring range was [0, 1]. The higher the score, the higher the content validity. After being scored by experts, the average validity score of each item and the average validity score of all items are >0.6, indicating high content validity.

The purpose is to reflect these more objective indicators, which more truly reflects the psychological load level of the students' vocal music class; and for those relatively vague indicators, such as the students' personal psychological characteristics, attention, emotion, will and other indicators, the method of fuzzy mathematics is used to evaluate, it can use accurate mathematics. Further construct validity analysis was carried out, using SPSS 22.0 for validity analysis, the calculated KMO value was 0.778 > 0.7, and the Bartlett sphericity test value was 0 <0.5, so it was suitable for factor analysis and further factor analysis.

### Mental expressiveness regulation

The psychological expressiveness questionnaire is designed based on the influencing factors obtained from the survey of vocal music teachers. It investigates the behavioral performance of students in this influencing factor. It includes 12 factors and is divided into 40 items. The 5-level Likert scale is designed, with items ranging from “very agree” to “very disagree,” scored as 1–5 points, and only one answer can be selected for each question. The number of psychometric data points cannot be less than the number of free parameters, otherwise the model and estimated parameters cannot be identified. The free parameter preflag(i,j) is the number of parameters to be estimated in the model, including path coefficients pretab(a,b), factor loadings, error term variances, etc. Second, we establish a measurement scale for each latent variable in the model. Usually, the variance gr(a) of the latent variable is set to 1, that is, the latent variable is standardized; it is also possible to set the load of any factor in the index variable of the latent variable to a constant (snr(a) is 1), that is, the factor tb(i) is fixed.


(7) $$\left\{ \begin{array}{l} preflag(a(i),a(j))-pretab(a,b)=0\;\\ {}^{gr(a-b)}{/}_{gr(a)-1}\to 1 \end{array}\right.$$

(8) $$\begin{array}{r} snr\left(a\right)-snv\left(b\right)dvdi-tb\left(i\right)di=\frac{tmn\left(i\right)di-\exp\left(i\right)}{1+tmn\left(i\right)di-\exp\left(i+1\right)} \end{array}$$

S(a) is the variance covariance matrix of the residual item tmn(i) of the structural model, and low(x) and high(x) are the measurement error covariance matrices of the exogenous observation index x and the endogenous observation index nmt(a), respectively. The main criteria for judging classification rules include speed, accuracy, interpretability and scalability.


(9) $$\begin{array}{c} pe(high(x),low(x))=\left[\begin{array}{c} e(lov(i))-e(-lov(i))\\ p(lov(i))+p(-lov(i)) \end{array}\right] \end{array}$$

(10) $$\{\begin{array}{c} tmn(a)+tmn(b)=(1+tb(a))*nmt(b)\\ tmn(a)-tmn(b)=(1-tb(a))*nmt(a) \end{array}$$

In a structural equation model, the estimated parameters should minimize the “gap” between the model's implied covariance matrix and the sample covariance matrix. This “gap” is a function of the model parameters and is called the fit function. There are several ways to define a fit function, each of which corresponds to a parameter estimation method. Generally, due to instrumental variables and the two-stage least squares method do not rely on iterative methods, although the speed is faster in estimating parameters, the error is larger.

In the multiple linear regression analysis, when there is a strong correlation between some independent variables in Figure 1, using the least squares method to estimate, there will be a phenomenon inconsistent with the professional, making the results difficult to explain, this phenomenon is called collinearity. At present, the commonly used methods to solve collinearity are partial regression, principal component regression and ridge regression, but they all have different degrees of defects in the interpretation of the results. Since the linear structure model can be regarded as being built on the basis of latent variables, when some independent variables in regression analysis have strong correlation, a common factor can be extracted from them, that is, a latent variable can be constructed to analyze them. In order to compare the results obtained by the other two evaluation methods more intuitively, the author converts the results obtained by the scale method into points based on the percentage system. Then assign the highest score to 100 and the lowest score to 0 (as in method 1, the scale contains 13 items).

**Figure 1:** Regression architecture of mental expressiveness.

### Psychological creation of vocal music teaching

Through the literature review of vocal music teaching psychology, it is concluded that in the existing research, a total of 54 factors have been proposed and studied, but some influencing factors play different roles in different studies. Several influencing factors are studied, and the influence model is assumed at the beginning of the research, and the research is often to verify whether the model is correct or not. The four questions are mainly to investigate the emotional state of students when learning vocal music content, including negative emotions in normal times and exams, and positive emotions in normal times.

This paper intends to use the decision tree algorithm in the classification rules to mine the potential relationship between the symptom self-rating scale SCL-90 and the basic information of vocal students, and use the Apriori algorithm in the association rule in Figure 2 to mine the symptom self-rating scale SCL. The interrelationship among the various psychological factors in the 190 provides a scientific basis for the management of mental health education. The three topics are mainly to investigate the students' intentions and behaviors to persevere in learning in their usual study, so as to determine whether they can persist in completing their own set of tasks.

**Figure 2:** Classification of vocal music teaching psychology.

The student's score in each secondary indicator is multiplied by the weight of the indicator, and then added. Multiplied by the weight of the first-level index to which the index belongs, it is the score of the student on the objective index of psychological load in vocal music class. After establishing a structural equation model based on the above psychological data to standardize the model, the regression coefficient parameters of the three observed variables are above 0.3. The ratio of the chi-square test value to the degrees of freedom is 0.944, the psychological data is low, and the significant probability value *p* = 0.389 > 0.05, so the null hypothesis is accepted, so it is assumed that the model can fit the observed psychological data. The CFI value is 1 > 0.9, the RMSEA value is 0, and the model fit is very good.

### Expression of mental health elements

The student questionnaire is mainly based on the psychological data obtained from the teacher's questionnaire, and the first-line vocal music teachers think that the factors that have a greater impact on the academic achievement of high school students' vocal music are selected, and the selected factors are used to prepare a student questionnaire.

Table 2 can extract six main factors, which are the same as when designing the questionnaire, and the cumulative load of six factors reaches 66.87%. Therefore, the validity of the preliminary survey is better. The CFI value is 0.894, which is <0.9, and RESEA = 0.106 > 0.08. And because the load factor coefficient 0.17 of the observed variable is much smaller than 0.5, the model is poor and the model needs to be revised. After inspection, it was found that the residuals in the model were correlated, so a new model was obtained after further revision of the model. Psychological data selection is a common psychological data processing method for psychological data analysis and mining in the early stage, and it is the first step of psychological data preprocessing. Due to the large scale of the original psychological data set, mining and analyzing all the psychological data sets will cost a lot of computing resources and computing cycles, so it is necessary to perform psychological data selection operations on the psychological data sets to reduce the impact on the results. Collecting and finding the information records in the psychological data set according to the mining project objectives can simplify the content of the psychological data, and also discover the internal relationship between attributes and the laws hidden behind the psychological data.

**Table 2:** Description of mental health elements.

**Element number value**	**Description texts**	**Main factors**	**Health ratio**
Factor a	Suitability	0.30	0.01
	Satisfaction	0.29	0.86
Factor b	Tolerance	0.24	0.43
	Concentration	0.27	0.49
Factor c	Activity	0.59	0.97
	Degree of realization	0.80	0.63

In order to better find the influencing factors in Figure 3 that have an impact on the academic achievement of high school students' vocal music, select the top 60% of the influencing factors that the survey respondents are relatively important or very important in the above statistical psychological data. The survey respondents of 12 factors including belief, achievement motivation, vocal interest, learning persistence, academic mood, learning motivation, learning strategy, class time, thinking style, educational expectation, and educational involvement accounted for more than 60% of all respondents. Then calculate the KMO value of the psychological data and find that its value is 0.403 <0.5, so it is not suitable for further factor analysis, indicating that the correlation of variables is poor. However, from the perspective of evaluation accuracy, the single use of the scale method will also use the objective scale method to evaluate the fuzzy factors that affect students' psychological load.

**Figure 3:** Internal links between attributes of mental health elements.

There are three types of “identification” of the model: (1) Insufficient identification type: when t > m(m + 1)/2, there are infinitely many sets of parameter solutions, that is, the solutions are uncertain not allowed. When performing a statistical analysis of a linear structural equation model in SAS or SPSS software, calculations are automatically stopped for “under-identified” models. (2) Exact identification type: when r = m(m + 1)/2, the solutions of all parameters are unique, the degree of freedom for checking the rationality of the model must be zero, and the value of z2 is also zero. At this time, although the model can be identified (parameter estimates can be obtained), it is impossible to judge whether the model is reasonable or not statistically. (3) Transition identification type: when f < m(m + 1)/2, the researcher can add different conditions to the parameters to be estimated, so that the obtained parameters meet the statistical requirements. Therefore, when identifying the model, it should be fitted with as few parameters as possible.

### Psychological emotion recognition in vocal music teaching

The Psychological and Emotional Questionnaire for Vocal Music Teaching is mainly based on the 54 influencing factors summarized above to investigate the opinions of vocal music teachers on the above-mentioned influencing factors. The questionnaire is designed in the form of a 5-level Likert scale. The questionnaire includes a total of 56 questions, including 54 questions about influencing factors. The psychological data preprocessing operations generally include: psychological data selection, psychological data cleaning, psychological data integration, psychological data specification and psychological data reduction. Through the preprocessing operation of the psychological data of Figure 4, the level of mining can be greatly improved and the time spent in analysis can be reduced.

**Figure 4:** The significance of psychological emotion recognition in vocal music teaching.

In modeling, the *p*-value in the unstandardized value represents the significance of the path between the observed variable and the latent variable, and the *p*-value is the ratio of the S.E. value to the C.R. value, where the C.R. value needs to >1.96. After running, it is found that only the C.R. value of the fifth question is >1.96, and the rest are <1.96, so they are not significant, so the above model is less suitable, that is, the learning belief cannot establish a structural equation model with the academic achievement of vocal music. The overall fitness chi-square test value is 8.678, the ratio of chi-square value to degrees of freedom is 2.170, *p* = 0.07 > 0.05, accepting the null hypothesis, GFI = 0.981, AGFI = 0.928, CFI = 0.965, RMSEA value is 0.082, close to 0.08, so the adaptability of the model is better. From the above model, it can be learned that vocal anxiety has a negative impact on academic achievement.

## Application and analysis of the vocal music teaching psychological model based on cultivation and interpretation of students' expressiveness

### Simulation of the mental health model of vocal music teaching

The survey on the mental health model of front-line vocal music was carried out in two ways: on-site paper questionnaire survey and online questionnaire. A total of 24 questionnaires were issued, two were discarded, the recovery rate was 100%, and the effective rate was 91.7%. The survey of students is carried out in the form of paper questionnaires, which are presided over by their class teachers to ensure the authenticity and validity of the questionnaires. A total of 175 questionnaires were distributed to the students, 175 were recovered and two were discarded. The recovery rate was 100% and the effective rate was 98.9%. By comprehensively analyzing multiple fitting indices, the fitting degree of the model is evaluated. The goodness-of-fit test indicators provided by different analysis software are different.

This method not only draws on the respective advantages of the two methods, but also makes up for their respective shortcomings. It not only highlights the intuitiveness of objective index evaluation, but also increases the accuracy of fuzzy subjective index evaluation, so as to achieve our research goals more accurately. Therefore, when the sample is large, it is necessary to refer to other evaluation indicators. In general, when NNFI is close to or >1, the model fits well; the smaller the root mean square error of the approximation (RMSEA), the better the fit. Generally, the model fits well when it is < 0.08.

The relationship in Figure 5 between the 90 scale and the 16PF personality factor questionnaire scores: (1) Pearson correlation analysis showed that the nine factors of the SCL-90 scale were related to the stability, persistence, courage, self-discipline and sensitivity in the 16PF questionnaire. There is a correlation between skepticism, anxiety and tension, that is, vocational students with better personality characteristics have fewer mental health problems. (2) Structural model analysis showed that the nine indicators measuring mental health can better represent mental health (standard regression coefficient > 0.757), the main factors are stability, perseverance, courage, self-discipline, anxiety and tension. From the measurement results of the factor scores of the 16PF questionnaire, it can be seen that the average scores of vocal students in terms of adaptation and anxiety (x) and cowardice and decisiveness (y) are lower than those of the norm group. For the norm group: the average score of introversion and extroversion is higher than the norm group, q is lower than the norm group in emotionality and serenity and alertness. (3) Although the average score of the group was no different from that of the norm population, those with a score >8 were lower than the norm population.

**Figure 5:** The level of mental health in vocal music teaching.

The Cronbach coefficient refers to the degree of homogeneity of the items of the subscales and the total scale. When judging the internal consistency of the scale, the number of scale items directly affects the reliability of the scale. If the number of items increases, the Cronbach will increase accordingly. On a scale of around 10 items, the Cronbach's score should be above 0.80. Psychological data cleaning is mainly to screen and remove duplicate psychological data, supplement and improve incomplete psychological data, and correct or delete erroneous psychological data. The repeated psychological data is mainly the information with the same attribute value in Figure 6, the incomplete psychological data is mainly the missing information, and the wrong data is mainly the information directly written into the psychological database without judgment.

**Figure 6:** Information on the mental health model of vocal music teaching.

There are 18 people who are relatively important and very important, accounting for 31.2%; 16 people, accounting for 32.3%, think that the factors of learning motivation are relatively important and very important; 17 people, accounting for 72.3%, think that the factors of learning strategy are relatively important and very important 37.3%; 16 people, accounting for 32.3%, think the thinking style is more important and very important, they think that the factors of family education expectations are more important and there are 14 people who are important, accounting for 31.3%; 16 people, accounting for 32.3%, think that the factors involved in education are relatively important and very important.

### Example application and analysis

The evaluation-related psychological data is derived from the vocal music student mental health evaluation system. The processing operation depends on the amount of psychological data. If the psychological data to be processed is relatively small, the null value can be filled according to the rules; if the data to be processed is relatively large, then you can find a value to fill in the empty value. Among them, 48 students who did not participate in the evaluation were excluded, and the psychological evaluation information of the students who participated in the evaluation met the research specifications. The establishment of a dimensional model is the basis for the realization of emotional computing, and it is also the basis for the machine to understand and respond to the learner's emotion based on the dimensional emotional prediction.

Among them, 86 students with many missing items are no longer available as research object. After psychological data cleaning, there are a total of 180 records that can be used for psychological data mining operations. From “serious” to “basically no impact,” it is scored on a scale of 1–5, and only one answer can be selected for each question. (1) The respondents are all teachers with more than 3 years of teaching experience, so they all have certain knowledge and opinions in vocal music teaching. The average age of the respondents is 35 years old, and the average teaching age is 11 years. Therefore, the respondents have their own reasons and abilities to judge the vocal music learning of high school students. (2) In the investigation of the influencing factors, the reliability of the psychological data of the questionnaire, the Cronbach's α reliability analysis coefficient is 0.946, so the reliability of the questionnaire is good, and the psychological data analysis can be continued.

Psychological data specification is a crucial link in the processing of psychological data mining. When processing the psychological data in Figure 7, it is first necessary to convert the data into a form of psychological data that conforms to psychological data mining. The conversion principle usually uses continuous psychological data discrete and discrete classification. For the structural equation model, after the model is operated, the *p*-value of the unstandardized coefficient needs to be < 0.05, so as to accurately track the evolution of emotional state and make up for the shortcomings of discrete emotion models. Psychology shows that the value of the emotional dimension depends on the cognitive behavior of the marker, such as memory and attention, and is highly subjective. It can be seen from the figure that after standardizing the model, the regression coefficient parameters are mostly above 0.5. After viewing the regression coefficient table, the *p*-values are all < 0.05, so the reliability of the questionnaire design is acceptable.

**Figure 7:** Student mental health assessment system data export assessment.

For the structural model, the degree of fit between the observed psychological data and the model is measured by the ratio of chi-square to degrees of freedom, GFI, AGFI, CFI, and RMSEA, where the ratio of chi-square to degrees of freedom must be <3; the value indicates the degree of similarity between the model and the observed psychological data, and if it is >0.9, it indicates that the similarity between the model and the observed psychological data is high; the RMSEA value measures the degree of dissimilarity between the model and the observed psychological data, preferably < 0.08, indicates the fit level of the model with the observed psychological data. The chi-square test value of the overall fitness of the model is 20.078, the ratio of chi-square value to degrees of freedom is 4.016, GFI = 0.953, AGFI = 0.859 <0.9, CFI = 0.887 <0.9, RMSEA value is 0.132 > 0.08, so the model is suitable. The degree of matching is poor, and the model needs to be further revised. The correction model needs to be carried out from the perspectives of observed variables and residuals. From the above two perspectives, the model is revised, in which errors in the system are found through the coefficient data, and a correlation path is added to obtain a new model.

## Conclusion

With the increasing maturity and wide application of psychological data mining technology, it has also been well used in vocal music teaching and management in colleges and universities. In this paper, by collecting and consulting relevant materials and literature, the psychological data mining technology in vocal music teaching is deeply studied and researched, and the psychological data mining technology is tried to be applied to the analysis of vocal music students' mental health data, so as to find out the hidden data of students' mental health information. The research order of this paper is as follows: firstly, search from the psychological database, screen out the existing researches on the influencing factors of middle school students' vocal academic achievement, and summarize the existing influencing factors from the above researches; secondly, based on the summed up influencing factors, take high school vocal music teachers as the object of investigation, and based on the obtained psychological data, summarize the factors that currently have an impact on the academic achievement of vocal music;. Finally, combined with the students' final vocal academic achievement, the research method of structural equation is used to analyze the relationship between students' vocal academic achievement and the factors that affect their vocal academic achievement. Structural model can filter errors and individual differences as much as possible; in addition to examining the direct effect between variables, it can also examine the indirect effect between variables at the same time. It is of practical significance to promote the reform of physical education, to check and improve the quality of teaching, and to speed up the management of teaching. It is sincerely hoped that this research will attract the attention of relevant educational administration departments and strengthen further research in this area.

## Data availability statement

The original contributions presented in the study are included in the article/supplementary material, further inquiries can be directed to the corresponding author/s.

## Author contributions

The author confirms being the sole contributor of this work and has approved it for publication.

## Conflict of interest

The author declares that the research was conducted in the absence of any commercial or financial relationships that could be construed as a potential conflict of interest.

## Publisher's note

All claims expressed in this article are solely those of the authors and do not necessarily represent those of their affiliated organizations, or those of the publisher, the editors and the reviewers. Any product that may be evaluated in this article, or claim that may be made by its manufacturer, is not guaranteed or endorsed by the publisher.

## References

[1] LianY. On the teaching reform methods of vocal music performance under the background of educational psychology. Psychiatr Danub. (2022) 34:511–3. Available online at: https://hrcak.srce.hr/277190

[2] YeY. Application of positive psychology in classroom teaching of vocal music. Revista Argentina de Clí*nica Psicológica*. (2020) 29:353. 10.24205/03276716.2020.48

[3] PunamäkiRLVänskäMQuotaSRPerkoKDiabSY. Vocal emotion expressions in infant-directed singing: the impact of war trauma and maternal mental health and the consequences on infant development. Infant Child Dev. (2020) 29:e2176. 10.1002/icd.2176

[4] BroomheadPSkidmoreJBEggettDLMillsMM. The effects of a teacher-directed preperformance routine on expressive performance mindset. Bull Council Res Music Educ. (2018) (215):57–74. 10.5406/bulcouresmusedu.215.0057

[5] NápolesJSilveyBAMontemayorM. The influences of facial expression and conducting gesture on college musicians' perceptions of choral conductor and ensemble expressivity. Int J Music Educ. (2021) 39:260–71. 10.1177/0255761420926665

[6] PattonLDJenkinsTSHowellGLKeithAR. Unapologetically Black creative educational experiences in higher education: a critical review. Rev Res Edu. (2022) 46:64–104. 10.3102/0091732X221084321

[7] McEvoyCASalvadorK. Aligning culturally responsive and trauma-informed pedagogies in elementary general music. Gen Music Today. (2020) 34:21–8. 10.1177/1048371320909806

[8] KoopsLHKuebelCR. Self-reported mental health and mental illness among university music students in the United States. Res Stud Music Educ. (2021) 43:129–43. 10.1177/1321103X19863265

[9] JääskeläinenT. Using a transcendental phenomenological approach as a model to obtain a meaningful understanding of music students' experienced workload in higher education. Int J Educ Arts. (2022) 23, 1–22. 10.26209/ijea23n6

[10] MontemayorMSilveyBA. Conductor expressivity affects evaluation of rehearsal instruction. J Res Music Educ. (2019) 67:133–52. 10.1177/0022429419835198

[11] PanYYSunXYDangYNChenaMWangLShenL. Effect of music intervention on depression in graduate students. Music Edu Res. (2021) 23:41–9. 10.1080/14613808.2020.184705834002549

[12] SandgrenM. Exploring personality and musical self-perceptions among vocalists and instrumentalists at music colleges. Psychol Music. (2019) 47:465–82. 10.1177/0305735618761572

[13] PilchPHArnesonC. Using recitative to teach expressive singing: an old idea made new. J Sing. (2018) 75:25–32. Available online at: link.gale.com/apps/doc/A573095359/HRCA?u=anon~bde65cb4&sid=googleScholar&xid=11a28f3f.

[14] Grindstaff E. Music From the Dark and Silence: Incorporating Deaf, Hard of Hearing, and Visually Impaired Students into the Music Education Classroom. ENCOMPASS (2020).

[15] Rosa-NapalFCMuñoz-CarrilPCGonzález-SanmamedMTabeayoIR. Musical expression in the training of future primary education teachers in Galicia. Int J Music Educ. (2021) 39:50–65. 10.1177/0255761420919566

[16] CliffordBNStockdaleLACoyneSMRaineyVBenitezVL. Speaking of state of mind: maternal mental health predicts children's home language environment and expressive language. J Child Lang. (2022) 49:469–85. 10.1017/S030500092100013133818326

[17] HeymanLPerkinsRAraújoLS. Examining the health and well-being experiences of singers in popular music. J Pop Music Educ. (2019) 3:173–201. 10.1386/jpme.3.2.173_1

[18] KnappRKnappZ. Musicals and the envoicing of mental illness and madness: from lady in the dark to man of La Mancha (and beyond). J Interdis Voice Stud. (2019) 4:209–23. 10.1386/jivs_00006_1

[19] ZhouZ. The influence of choral practices and passive listening to music on creative thinking. Think Skills Creat. (2021) 42:100972. 10.1016/j.tsc.2021.100972

[20] JohnsonKHeiderscheitAA. Survey of music therapy methods on adolescent inpatient mental health units. J Music Ther. (2018) 55:463–88. 10.1093/jmt/thy01530339184

[21] KoziiOUlianovaVBilostotskaOKachmarOBakhmatNProkopchukV. Experience in developing imaginative and intonational competencies in future music teachers. Revista Romaneasca Pentru Educatie Multidimensionala. (2020) 12:16–37. 10.18662/rrem/12.4/331

[22] MartinecJ. The virtual choir: examining the benefits and obstacles of online teaching in the choral setting. Can Music Educ. (2020) 61:41–6.

[23] BremmerMNijsL. The role of the body in instrumental and vocal music pedagogy: a dynamical systems theory perspective on the music teacher's bodily engagement in teaching and learning. Front Educ. (2020) 5:79. 10.3389/feduc.2020.00079

[24] CzajkowskiAMLGreasleyAEAllisM. Mindfulness for musicians: a mixed methods study investigating the effects of 8-week mindfulness courses on music students at a leading conservatoire. Music Sci. (2020) 26:102970. 10.1177/1029864920941570

